The article "High-quality draft genome sequence and description of Haemophilus massiliensis sp. nov" was retracted in 2025. Reason: lack of ethics approval or compliance.

# High-quality draft genome sequence and description of *Haemophilus massiliensis* sp. nov.

**DOI:** 10.1186/s40793-016-0150-1

**Published:** 2016-04-14

**Authors:** Cheikh Ibrahima Lo, Senthil Alias Sankar, Bécaye Fall, Bissoume Sambe-Ba, Silman Diawara, Mamadou Wague Gueye, Oleg Mediannikov, Caroline Blanc-Tailleur, Boubacar Wade, Didier Raoult, Pierre-Edouard Fournier, Florence Fenollar

**Affiliations:** Aix-Marseille Université, URMITE, UM63, CNRS 7278, IRD 198, Inserm U1095, Faculté de médecine, Marseille, France; Campus international UCAD-IRD, Dakar, Senegal; Hôpital Principal, Dakar, Senegal; Special Infectious Agents Unit, King Fahd Medical Research Center, King Abdulaziz University, Jeddah, Saudi Arabia

**Keywords:** *Haemophilus massiliensis*, Genome, Taxono-genomics, Culturomics

## Abstract

Strain FF7^T^ was isolated from the peritoneal fluid of a 44-year-old woman who suffered from pelvic peritonitis. This strain exhibited a 16S rRNA sequence similarity of 94.8 % 16S rRNA sequence identity with *Haemophilus parasuis*, the phylogenetically closest species with a name with standing in nomenclature and a poor MALDI-TOF MS score (1.32 to 1.56) that does not allow any reliable identification. Using a polyphasic study made of phenotypic and genomic analyses, strain FF7^T^ was a Gram-negative, facultatively anaerobic rod and member of the family *Pasteurellaceae*. It exhibited a genome of 2,442,548 bp long genome (one chromosome but no plasmid) contains 2,319 protein-coding and 67 RNA genes, including 6 rRNA operons. On the basis of these data, we propose the creation of *Haemophilus massiliensis* sp. nov. with strain FF7^T^ (= CSUR P859 = DSM 28247) as the type strain.

**Electronic supplementary material:**

The online version of this article (doi:10.1186/s40793-016-0150-1) contains supplementary material, which is available to authorized users.

## Introduction

The genus *Haemophilus* (Winslow et al. 1917) was described in 1917 [1] and currently meningitis, bacteremia, sinusitis, and/or pneumonia [2].

The current taxonomic classification of prokaryotes relies on a combination of phenotypic and genotypic characteristics [3, 4]; including 16S rRNA sequence similarity, G + C content and DNA-DNA hybridization. However, these tools suffer from various drawbacks, mainly due to their threshold values that are not applicable to all species or genera [5, 6]. With the development of cost-effective, high-throughput sequencing techniques, dozens of thousands of bacterial genome sequences have been made available in public databases [7]. Recently, we developed a strategy named taxono-genomics in which genomic and phenotypic characteristics, notably the MALDI-TOF-MS spectrum, are systematically compared to the phylogenetically-closest species with a name with standing in nomenclature [8, 9].

The article "High-quality draft genome sequence and description of Haemophilus massiliensis sp. nov" was retracted in 2025. Reason: lack of ethics approval or compliance.

The strain FF7^T^ was isolated from the peritoneal fluid of a Senegalese woman suffering from pelvic peritonitis complicating a ruptured ovarian abscess. She was admitted to Hôpital Principal in Dakar, Senegal. *Haemophilus massiliensis* is a Gram-negative, facultatively anaerobic, oxidase and catalase-positive and non-motile rod shaped bacterium. This microorganism was cultivated as part of the MALDI-TOF-MS implementation in Hôpital Principal in Dakar, aiming at improving the routine laboratory identification of bacterial strains in Senegal [10].

Here, we present a summary classification and a set of features for *Haemophilus massiliensis* sp. nov. together with the description of the complete genome sequencing and annotation. These characteristics support the circumscription of the species *Haemophilus massiliensis*.

## Organism information

### Classification and features

In June 2013, a bacterial strain (Table 1) was isolated by cultivation on 5 % sheep blood-enriched Columbia agar (BioMérieux, Marcy l'Etoile, France) of a peritoneal fluid specimen obtained from a 44-year-old Senegalese woman who suffered from pelvic peritonitis that had complicated a ruptured ovarian abscess [10] and hospitalized in Hôpital Principal de Dakar, Senegal. The strain could not be identified using MALDI-TOF-MS. Strain FF7^T^ exhibited a 94.8 % 16S rRNA sequence identity with *Haemophilus parasuis* strain ATCC 19417^T^ (GenBank accession number AY362909), the phylogenetically-closest bacterial species with a validly published name (Fig. 1). These values were lower than the 98.7 % 16S rRNA gene sequence threshold recommended by Meier-Kolthoff et al., 2013 to delineate a new species within phylum *Proteobacteria* without carrying out wet lab or digital DNA-DNA hybridization [11].

**Table 1:** Classification and general features of *Haemophilus massiliensis* strain FF7^T^ [13]

MIGS ID	Property	Term	Evidence code^a^
	Current classification	Domain: *Bacteria*	TAS [26]
		Phylum: *Proteobacteria*	TAS [27]
		Class: *Gammaproteobacteria*	TAS [28, 29]
		Order: *Pasteurellales*	TAS [29, 30]
		Family: *Pasteurellaceae*	TAS [31, 32]
		Genus: *Haemophilus*	TAS [1, 33]
		Species: *Haemophilus massiliensis*	IDA
		Type strain: FF7^T^	IDA
	Gram stain	Negative	IDA
	Cell shape	Rod	IDA
	Motility	Not motile	IDA
	Sporulation	Non-spore forming	IDA
	Temperature range	Mesophile	IDA
	Optimum temperature	37 °C	IDA
	pH range; Optimum	7.2-7.4; 7.3	
	Carbon source	Unknown	NAS
	Energy source	Unknown	NAS
MIGS-6	Habitat	Human peritoneal fluid	IDA
MIGS-6.3	Salinity	Unknown	
MIGS-22	Oxygen requirement	Facultatively anaerobic	IDA
MIGS-15	Biotic relationship	Free living	IDA
MIGS-14	Pathogenicity	Unknown	
	Biosafety level	2	
	Isolation	Human	IDA
MIGS-4	Geographic location	Senegal	IDA
MIGS-5	Sample collection time	June 2013	IDA
MIGS-4.1	Latitude	14° 40' N	IDA
MIGS-4.1	Longitude	17° 26' W	IDA
MIGS-4.3	Depth	Surface	IDA
MIGS-4.4	Altitude	12 m above sea level	IDA

^a^Evidence codes - IDA: Inferred from Direct Assay; TAS: Traceable Author Statement (i.e., a direct report exists in the literature); NAS: Non-traceable Author Statement (i.e., not directly observed for the living, isolated sample, but based on a generally accepted property for the species, or anecdotal evidence). These evidence codes are from the Gene Ontology project [34]. If the evidence is IDA, then the property was directly observed for a live isolate by one of the authors or an expert mentioned in the acknowledgements

The article "High-quality draft genome sequence and description of Haemophilus massiliensis sp. nov" was retracted in 2025. Reason: lack of ethics approval or compliance.

**Fig. 1:** Phylogenetic tree showing the position of *Haemophilus massiliensis* strain FF7^T^ relative to the most closely related type strains other type strains (type = ^T^) within the genus *Haemophilus*. The GenBank accession numbers for 16S rRNA genes are indicated in parentheses. An asterisk marks strains that have a genome sequence in the NCBI database. Sequences were aligned using MUSCLE [35], and a phylogenetic tree inferred using the Maximum Likelihood method with Kimura 2-parameter model using the MEGA software. Numbers at the nodes are percentages of bootstrap values obtained by repeating the analysis 1,000 times to generate a majority consensus tree. Only bootstrap values equal to or greater than 70 % are displayed. The scale bar represents a rate of substitution per site of 1 %. *Escherichia coli* strain ATCC 11775^T^ was used as outgroup

Different growth temperatures (25 °C, 30 °C, 37 °C, 45 °C, and 56 °C) were tested. Growth was obtained between 25 and 45 °C, with the optimal growth temperature being 37 °C. Colonies were 0.5 mm in diameter and non-hemolytic on 5 % sheep blood-enriched Columbia agar (BioMérieux). Gram staining showed rod-shaped Gram-negative bacilli that were not motile and unable to form spores (Fig. 2). In electron microscopy, cells had a mean length of 2.6 μm (range 2.0-3.2 μm) and width of 0.35 μm (range 0.2-0.5 μm) (Fig. 2). Growth of the strain was tested under anaerobic and microaerophilic conditions using GENbag anaer and GENbag microaer systems, respectively (BioMérieux), and under aerobic conditions, with or without 5 % CO_2_. Optimal growth was observed at 37 °C under aerobic and microaerophilic conditions. Strain FF7^T^ exhibited oxidase and catalase activities. Using an API ZYM strip (BioMérieux), positive reactions were observed for acid phosphatase, leucine arylamidase, esterase, alkaline phosphatase and Naphthol-AS-BI-phosphohydrolase. Negative reactions were noted for α-chymotrypsin, cystine arylamidase, valine arylamidase, trypsin, α-glucosidase, β- glucosidase, esterase-lipase, leucine arylamidase, α-galactosidase, β-galactosidase, β-glucuronidase, α-mannosidase, α-fucosidase, and N-acetyl-β-glucosaminidase. Using API 20NE (BioMérieux), positive reactions were obtained for L-arginine, esculin, ferric citrate and urea but negative reactions were observed for D-glucose, L-arabinose, D-maltose, D-mannose, D-mannitol, potassium gluconate and N-acetyl-glucosamine. *Haemophilus**massiliensis* strain FF7^T^ is susceptible to penicillin, amoxicillin, amoxicillin/clavulanic acid, imipenem, gentamicin, ceftriaxone and doxycycline but resistant to vancomycin, nitrofurantoin, and trimethoprim/sulfamethoxazole. The minimum inhibitory concentrations for some antibiotics tested with *Haemophilus**massiliensis* strain FF7^T^ sp. nov. are listed in Additional file 1: Table S1. Five species validly published names in the *Haemophilus* genus were selected to make a phenotypic comparison with our new species named *Haemophilus**massiliensis* detailed in Additional file 2: Table S2.

The article "High-quality draft genome sequence and description of Haemophilus massiliensis sp. nov" was retracted in 2025. Reason: lack of ethics approval or compliance.

**Fig. 2:** Morphology of *Haemophilus massiliensis* sp. nov. strain FF7^T^. **a**: Gram staining. **b**: Transmission electron microscopy. The scale bar represents 500 nm

MALDI-TOF protein analysis was carried out as previously described [12] using a Microflex LT (Bruker Daltonics, Leipzig, Germany). For strain FF7^T^, scores ranging from 1.32 to 1.56 were obtained with spectra available in the Brüker database. Therefore the isolate could not be classified within any known species. The reference mass spectrum from strain FF7^T^ was incremented in our database (Additional file 3: Figure S1). Finally, the gel view showed that all members of the genus *Haemophilus* for which spectra were available in the database could be discriminated (Additional file 4: Figure S2).

## Genome sequencing information

### Genome project history

The strain was selected for sequencing on the basis of its 16S rRNA similarity, phylogenetic position, and phenotypic differences with other members of the genus *Haemophilus*, and is part of a study aiming at using MALDI-TOF-MS for the routine identification of bacterial isolates in Hôpital Principal in Dakar [10]. It is the eleventh genome of a *Haemophilus* species and the first genome of *Haemophilus massiliensis* sp. nov. The Genbank accession number is CCFL00000000 and consists of 46 contigs. Table 2 shows the project information and its association with MIGS version 2.0 compliance [13].

The article "High-quality draft genome sequence and description of Haemophilus massiliensis sp. nov" was retracted in 2025. Reason: lack of ethics approval or compliance.

**Table 2:** Project information

MIGS ID	Property	Term
MIGS-31	Finishing quality	High-quality draft
MIGS-28	Libraries used	Mate-Pair 3.1 kb library
MIGS-29	Sequencing platforms	Illumina Miseq
MIGS-31.2	Fold coverage	42.54
MIGS-30	Assemblers	CLC GENOMICSWB4
MIGS-32	Gene calling method	Prodigal
	Locus Tag	Not indicated
	Genbank ID	CCFL00000000
	Genbank Date of Release	August 22, 2014
	GOLD ID	Ga0059233
	BIOPROJECT	PRJEB5521
MIGS-13	Source material identifier	CSUR P859, DSM 28247
	Project relevance	MALDI-TOF-MS implementation in Dakar

### Growth conditions and genomic DNA preparation

*Haemophilus massiliensis* sp. nov., strain FF7^T^ (= CSUR P859= DSM 28247) was grown aerobically on 5 % sheep blood-enriched Columbia agar (BioMérieux) at 37 °C. Bacteria grown on four Petri dishes were resuspended in 5x100 μL of TE buffer; 150 μL of this suspension was diluted in 350 μL TE buffer 10X, 25 μL proteinase K and 50 μL sodium dodecyl sulfate for lysis treatment. This preparation was incubated overnight at 56 °C. Extracted DNA was purified using 3 successive phenol-chloroform extractions and ethanol precipitations. Following centrifugation, the DNA was suspended in 65 μL EB buffer. The genomic DNA (gDNA) concentration was measured at 14.7 ng/μl using the Qubit assay with the high sensitivity kit (Life Technologies, Carlsbad, CA, USA).

### Genome sequencing and assembly

Genomic DNA of *Haemophilus massiliensis* FF7^T^ was sequenced on the MiSeq sequencer (Illumina, San Diego, CA, USA) with the Mate-Pair strategy. The gDNA was barcoded in order to be mixed with 11 other projects with the Nextera Mate-Pair sample prep kit (Illumina). The Mate-Pair library was prepared with 1 μg of genomic DNA using the Nextera Mate-Pair Illumina guide. The gDNA sample was simultaneously fragmented and tagged with a Mate-Pair junction adapter. The pattern of the fragmentation was validated on an Agilent 2100 BioAnalyzer (Agilent Technologies, Santa Clara, CA, USA) with a DNA 7500 labchip. The DNA fragments ranged in size from 1 kb up to 10 kb with an optimal size at 4.08 kb. No size selection was performed and only 464 ng of tagmented fragments were circularized. The circularized DNA was mechanically sheared to small fragments with an optimal at 569 bp on the Covaris S2 device in microtubes (Covaris, Woburn, MA, USA). The library profile was visualized on a High Sensitivity Bioanalyzer LabChip (Agilent Technologies) and the final library concentration was measured at 24.42 nmol/L. The libraries were normalized at 2nM and pooled. After a denaturation step and dilution at 15 pM, the pool of libraries was loaded onto the reagent cartridge and then onto the instrument along with the flow cell. Automated cluster generation and sequencing run were performed in a single 39-h-run in a 2x251-bp. Total information of 10.1Gb was obtained from a 1,189 K/mm2 cluster density with a cluster passing quality control filters of 99.1 % (22,579,000 clusters). Within this run, the index representation for *Haemophilus massiliensis* was 9.72 %. The 1,976,771 paired reads were filtered according to the read qualities. These reads were trimmed, then assembled using the CLC genomicsWB4 software. Finally, the draft genome of *Haemophilus**massiliensis* consists of 9 scaffolds with 46 contigs and generated a genome size of 2.4 Mb with a 46.0 % G + C content.

The article "High-quality draft genome sequence and description of Haemophilus massiliensis sp. nov" was retracted in 2025. Reason: lack of ethics approval or compliance.

### Genome annotation

Open Reading Frames were predicted using Prodigal [14] with default parameters but the predicted ORFs were excluded if they spanned a sequencing gap region. The predicted bacterial protein sequences were searched against the GenBank database [15] and the Clusters of Orthologous Groups databases using BLASTP. The tRNAScanSE tool [16] was used to find tRNA genes, whereas ribosomal RNAs were found using RNAmmer [17] and BLASTn against the GenBank database. Lipoprotein signal peptides and the number of transmembrane helices were predicted using SignalP [18] and TMHMM [19] respectively. ORFans were identified if their BLASTP E-value was lower than 1e-03 for alignment length greater than 80 amino acids. If alignment lengths were smaller than 80 amino acids, we used an E-value of 1e-05. Such parameter thresholds have already been used in previous works to define ORFans. Artemis [20] was used for data management and DNA Plotter [21] for visualization of genomic features. The Mauve alignment tool (version 2.3.1) was used for multiple genomic sequence alignment [22]. To estimate the mean level of nucleotide sequence similarity at the genome level, we used the AGIOS home-made software [9]. Briefly, this software combines the Proteinortho software [23] for detecting orthologous proteins in pairwise genomic comparisons, then retrieves the corresponding genes and determines the mean percentage of nucleotide sequence identity among orthologous ORFs using the Needleman-Wunsch global alignment algorithm. The script created to calculate AGIOS values was named MAGi and is written in perl and bioperl modules. GGDC analysis was also performed using the GGDC web server as previously reported [24, 25].

## Genome properties

The genome of *Haemophilus**massiliensis* strain FF7^T^ is 2,442,548 bp-long with a 46.0 % G + C content. Of the 2,386 predicted genes, 2,319 were protein- coding genes and 67 were RNA genes, including six complete rRNA operons. A total of 1,885 genes (79.5 %) were assigned a putative function. A total of 36 genes were identified as ORFans (1.5 %). The remaining genes were annotated as hypothetical proteins. The properties and statistics of the genome are summarized in Table 3 and Fig. 3. The distribution of genes into COGs functional categories is presented in Table 4 and Fig. 4. The distribution of genes into COGs categories was similar for most of the compared species (Fig. 4). However, *H. influenzae* and *H. aegyptius* were over-represented for category N (cell motility), and *H. ducreyi* was under-represented for category W (extracellular structures) (Fig. 4).

The article "High-quality draft genome sequence and description of Haemophilus massiliensis sp. nov" was retracted in 2025. Reason: lack of ethics approval or compliance.

**Table 3:** Genome statistics

Attribute	Value	% of total^a^
Genome size (bp)	2,442,548	100
DNA coding (bp)	2,181,795	89.35
DNA G + C (bp)	1,123,572	46.0
DNA scaffolds	46	-
Total genes	2,386	100
Protein coding genes	2,319	97.19
RNA genes	67	2.80
Pseudo genes	N/D^b^	-
Gens in internal clusters	N/D^b^	-
Genes with function prediction	1,885	79.00
Genes assigned to COGs	2,093	87.72
Genes with Pfam domains	1,419	59.47
Genes with signal peptides	188	7.87
Genes with transmembrane helices	445	18.65
ORFan genes	36	1.50
CRISPR repeats	2	0.08

^a^The total is based on either the size of the genome in base pairs or the total number of protein coding genes in the annotated genome

^b^N/D = not determined

**Fig. 3:** Graphical circular map of the *Haemophilus massiliensis* strain FF7^T^ chromosome. From the outside in, the outer two circles show open reading frames oriented in the forward (colored by COG categories) and reverse (colored by COG categories) directions, respectively. The third circle marks the tRNA genes (green). The fourth circle shows the G + C% content plot. The inner-most circle shows GC skew, purple indicating negative values whereas olive for positive values

**Table 4:** Number of genes associated with general COG functional categories

Code	Value	% of total^a^	Description
J	160	6.90	Translation
A	1	0.04	RNA processing and modification
K	150	6.47	Transcription
L	131	5.65	Replication, recombination and repair
B	0	0	Chromatin structure and dynamics
D	28	1.21	Cell cycle control, mitosis and meiosis
V	37	1.60	Defense mechanisms
T	46	1.98	Signal transduction mechanisms
M	135	5.82	Cell wall/membrane biogenesis
N	6	0.26	Cell motility
W	9	0.39	Extracellular structures
U	58	2.50	Intracellular trafficking and secretion
O	109	4.70	Posttranslational modification, protein turnover, chaperones
C	163	7.03	Energy production and conversion
G	228	9.83	Carbohydrate transport and metabolism
E	234	10.09	Amino acid transport and metabolism
F	63	2.72	Nucleotide transport and metabolism
H	117	5.05	Coenzyme transport and metabolism
I	62	2.67	Lipid transport and metabolism
P	152	6.55	Inorganic ion transport and metabolism
Q	34	1.47	Secondary metabolites biosynthesis, transport and catabolism
R	258	11.13	General function prediction only
S	174	7.50	Function unknown
-	226	9.53	Not in COGs

^a^The total is based on the total number of protein coding genes in the annotated genome

The article "High-quality draft genome sequence and description of Haemophilus massiliensis sp. nov" was retracted in 2025. Reason: lack of ethics approval or compliance.

**Fig. 4:** Distribution of functional classes of predicted genes in the genomes from *Haemophilus massiliensis* (HM) strain FF7^T^, *H. parasuis* (HPA) strain ATCC 19417^T^, *Aggregatibacter segnis* (AE) strain ATCC 33393^T^, *H. aegyptius* (HA) strain ATCC 11116^T^, *H. ducreyi* (HD) strain CIP 54.2, *H. haemolyticus* (HH) strain ATCC 33390^T^, *H. influenzae* (HI) strain ATCC 33391^T^, *H. parahaemolyticus* (HP), *H. parainfluenzae* (HPI) strain ATCC 10014^T^, *H. pittmaniae* (HPT) strain HK 85^T^, and *H. sputorum* (HS) strain CCUG 13788^T^ chromosomes according to the clusters of orthologous groups of proteins

## Insights from the genome sequence

Here, we compared the genome sequences of *Haemophilus**massiliensis* strain FF7^T^ (GenBank accession number CCFL00000000) with those of *Haemophilus parasuis* strain SH0165 (CP001321), *Haemophilus influenzae* strain Rd KW20 (L42023), *Aggregatibacter segnis* strain ATCC 33393^T^ (AEPS00000000), *Haemophilus sputorum* strain CCUG 13788^T^ (AFNK00000000), *Haemophilus pittmaniae* strain HK 85 (AFUV00000000), *Haemophilus aegyptius* strain ATCC 1111^T^ (AFBC00000000), *Haemophilus parainfluenzae* strain ATCC 33392^T^ (AEWU00000000), *Haemophilus haemolyticus* strain M21621 (AFQQ00000000), *Haemophilus ducreyi* strain 35000HP (AE017143), and *Haemophilus parahaemolyticus* strain HK385 (AJSW00000000).

The draft genome of *Haemophilus massiliensis* has a larger size than that of *H. parasuis*, *H. influenzae**,**A. segnis*, *H. sputorum*, *H. pittmaniae*, *H. aegyptius*, *H. parainfluenzae*, *H. haemolyticus*, *H. ducreyi*, and *H. parahaemolyticus* (2.44, 2.27, 1.83, 1.99, 2.14, 2.18, 1.92, 2.11, 2.09, 1.7, and 2.03 Mb, respectively). The G + C content of *Haemophilus massiliensis* is higher than those of *H. parasuis*, *H. influenzae**,**A. segnis*, *H. sputorum*, *H. pittmaniae*, *H. aegyptius*, *H. parainfluenzae*, *H. haemolyticus**,**H. ducreyi*, and *H. parahaemolyticus* (46.0, 40.0, 38.2, 42.5, 39.7, 42.5, 38.1, 39.1, 38.4, 38.2, and 40.1 %, respectively). As it has been suggested in the literature that the G + C content deviation is at most 1 % within species, these data are an additional argument for the creation of a new taxon [25].

The gene content of *Haemophilus massiliensis* is larger than those of *H. parasuis**,**H. influenzae**,**A. segnis*, *H. sputorum*, *H. aegyptius**,**H. parainfluenzae*, *H. haemolyticus*, *H. ducreyi*, and *H. parahaemolyticus* (2,319, 2,299, 1,765, 1,956, 2,072, 2,020, 2,068, 2,056, 1,717, and 1,980, respectively) but smaller than that of *H. pittmaniae* (2,390). However the distribution of genes into COG categories was similar in all compared genomes as shown in Fig. 4. In addition, in this last figure, *Haemophilus**massiliensis* shared 2,021, 1,956, 2,020, 1,717, 1,977, 1,610, 1,980, 2,010, 2,390, and 2,123 orthologous genes with *H. parasuis*, *A. segnis*, *H. aegyptius*, *H. ducreyi**,**H. haemolyticus*, *H. influenzae*, *H. parahaemolyticus**,**H. parainfluenzae*, *H. pittmaniae*, and *H. sputorum*, respectively (Table 5). Among species with standing in nomenclature, AGIOS values ranged from 71.19 between *H. pittmaniae* and *H. ducreyi* to 97.31 % between *H. influenzae* and *H. aegyptius*. When compared to other species, *Haemophilus**massiliensis* exhibited AGIOS values ranging from 70.00 with *H. ducreyi* to 74.19 with *A. segnis*. We obtained similar results using the GGDC software, as dDDH values ranged from 0.201 to 0.777 between studied species, and were 0.248 between *Haemophilus massiliensis* and *Haemophilus parasuis*. These values confirm the status of *Haemophilus massiliensis* as a new species.

The article "High-quality draft genome sequence and description of Haemophilus massiliensis sp. nov" was retracted in 2025. Reason: lack of ethics approval or compliance.

**Table 5:** dDDH values (upper right) and AGIOS values obtained (lower left)

	HM^a^	HPA^b^	HI^c^	HA^d^	AE^e^	HH^f^	HP^g^	HD^h^	HS^i^	HPT^j^	HPH^k^
HM	**2,319**	0.248	0.222	0.203	0.204	0.202	0.243	0.285	0.232	0.235	0.201
HPA	70.64	**2,021**	0.296	0.292	0.244	0.278	0.236	0.237	0.262	0.283	0.251
HI	72.76	72.75	**1,610**	0.777	0.234	0.433	0.259	0.252	0.279	0.252	0.239
HA	72.80	72.67	97.31	**2,020**	0.231	0.434	0.237	0.244	0.271	0.242	0.235
AE	74.19	71.93	75.72	75.69	**1,956**	0.235	0.243	0.267	0.255	0.246	0.232
HH	72.72	72.64	91.85	91.80	75.72	**1,977**	0.240	0.250	0.284	0.247	0.246
HP	70.16	75.40	74.07	73.98	71.97	73.79	**1,980**	0.239	0.218	0.293	0.227
HD	70.00	74.81	72.47	72.36	71.34	72.33	75.34	**1,717**	0.228	0.270	0.251
HS	70.23	75.06	73.46	73.39	72.33	73.54	78.00	75.68	**2,123**	0.319	0.280
HPT	72.55	71.51	76.38	76.48	74.95	76.64	71.88	71.19	72.88	**2,390**	0.269
HPH	72.67	72.71	79.69	79.70	76.20	79.96	73.36	72.30	74.14	78.94	**2,010**

The values printed in bold are gene numbers. Digital DDH similarities between the genomes were calculated using GGDC web server version 2.0. under recommend setting [36, 37]; formula 2 is recommended, particularly for draft genomes. ^a^ *Haemophilus massiliensis*, ^b^ *Haemophilus parasuis*, ^c^ *Haemophilus influenzae*, ^d^ *Haemophilus aegyptius*, ^e^ *Aggregatibacter segnis*, ^f^ *Haemophilus haemolyticus*, ^g^ *Haemophilus parainfluenzae*, ^h^ *Haemophilus ducreyi*, ^i^ *Haemophilus sputorum*, ^j^ *Haemophilus pittmaniae* and ^k^ *Haemophilus parahaemolyticus*

The article "High-quality draft genome sequence and description of Haemophilus massiliensis sp. nov" was retracted in 2025. Reason: lack of ethics approval or compliance.

## Conclusions

On the basis of phenotypic, phylogenetic and genomic analyses, we formally propose the creation of *Haemophilus massiliensis* sp. nov. that contains strain FF7^T^ (CSUR P859 = DSM 28247) which is the type strain The strain was isolated from a peritoneal fluid specimen from a 44-year-old Senegalese woman admitted to Hôpital Principal in Dakar, Senegal.

## Description of *Haemophilus massiliensis* sp. nov.

*Haemophilus massiliensis* (mas.il.i.en’sis. L. gen. masc. n. massiliensis, of *Massilia*, the Latin name of Marseille where strain FF7^T^ was characterized).

*Haemophilus massiliensis* is a facultatively anaerobic Gram-negative bacterium, non-endospore forming and non-motile. Colonies are not haemolytic, round, and light with a size of 0.5-1 mm on blood-enriched Colombia agar. Cells are rod-shapped with a mean length of 2.6 μm (range 2.0-3.2 μm) and a mean diameter of 0.35 μm (range 0.2-0.5 μm). Growth occurs between 25 and 45 °C, with optimal growth occurring at 37 °C. Catalase and oxidase reactions are positive. Positive reactions are also observed for acid phosphatase, leucine arylamidase, esterase, alkaline phosphatase, Naphthol-AS-BI-phosphohydrolase, L-arginine, esculin, ferric citrate, and urea. *Haemophilus**massiliensis* strain FF7^T^ is susceptible to penicillin, amoxicillin, amoxicillin/clavulanic acid, imipenem, gentamicin, ceftriaxone and doxycycline but resistant to vancomycin, nitrofurantoin and trimethoprim/sulfamethoxazole.

The type strain is FF7^T^ (= CSUR P859 = DSM 28247) and was isolated from the peritoneal fluid of a 44-year-old Senegalese woman suffering from pelvic peritonitis in Dakar, Senegal.

## Additional files

Additional file 1: Table S1. Antimicrobial susceptibility and minimum inhibitory concentrations (MIC) of Haemophilus massiliensis strain FF7T sp nov. (DOC 30 kb) Additional file 2: Table S2. Differential characteristics of Haemophilus massiliensis strain FF7T (data from this study), H. influenzae strain ATCC 33391T [1, 33], H. sputorum strain CCUG 13788T [38, 39], H. pittmaniae strain HK 85T [40, 41], Haemophilus felis strain TI189T [42, 43] and H. parasuis strain ATCC 19417T [33, 41]. na = data not available. (DOC 57 kb) Additional file 3: Figure S1. Reference mass spectrum from *Haemophilus massiliensis* strain FF7^T^. Spectra from 12 individual colonies were compared and a reference spectrum was generated. (DOCX 25 kb) Additional file 4: Figure S2. Gel view comparing *Haemophilus massiliensis* strain FF7^T^ to the members of the *Haemophilus* genus*.* The gel view displays the raw spectra of all loaded spectrum files arranged in a pseudo-gel like look. The x-axis records the m/z value. The left y-axis displays the running spectrum number originating from subsequent spectra loading. The peak intensity is expressed by a Gray scale scheme code. The color bar and the right y-axis indicate the relation between the color a peak is displayed with and the peak intensity in arbitrary units. Displayed species are indicated on the left. (DOCX 192 kb)

The article "High-quality draft genome sequence and description of Haemophilus massiliensis sp. nov" was retracted in 2025. Reason: lack of ethics approval or compliance.

## Abbreviations

CSUR: Strains collection of *Rickettsia* Unit
CNERS: National Ethics Committee of Senegal
MALDI-TOF MS: Matrix-assisted laser-desorption/ionization time-of-flight mass spectrometry
MAGi: Marseille Average genomic identity
dDDH: digital DNA-DNA hybridization
URMITE: Unit of Research on Emergent Infectious and Tropical Diseases
